# Autonomous glucose metabolic reprogramming of tumour cells under hypoxia: opportunities for targeted therapy

**DOI:** 10.1186/s13046-020-01698-5

**Published:** 2020-09-14

**Authors:** Mingyao Huang, Liang Yang, Xueqiang Peng, Shibo Wei, Qing Fan, Shuo Yang, Xinyu Li, Bowen Li, Hongyuan Jin, Bo Wu, Jingang Liu, Hangyu Li

**Affiliations:** Department of General Surgery, the Fourth Affiliated Hospital, China Medical University, Shenyang, 110032 China

**Keywords:** Hypoxia, Tumour, Glucose, Metabolic reprogramming

## Abstract

Molecular oxygen (O_2_) is a universal electron acceptor that is eventually synthesized into ATP in the mitochondrial respiratory chain of all metazoans. Therefore, hypoxia biology has become an organizational principle of cell evolution, metabolism and pathology. Hypoxia-inducible factor (HIF) mediates tumour cells to produce a series of glucose metabolism adaptations including the regulation of glucose catabolism, glycogen metabolism and the biological oxidation of glucose to hypoxia. Since HIF can regulate the energy metabolism of cancer cells and promote the survival of cancer cells, targeting HIF or HIF mediated metabolic enzymes may become one of the potential treatment methods for cancer. In this review, we summarize the established and recently discovered autonomous molecular mechanisms that can induce cell reprogramming of hypoxic glucose metabolism in tumors and explore opportunities for targeted therapy.

## Background

Hypoxia is a characteristic feature of locally advanced solid tumours resulting from an imbalance in oxygen (O_2_) supply and consumption in the proximity [1]. The disordered vasculature that is developed in response to the oxygen demand of rapidly growing tumours leads to widespread hypoxic regions in solid tumours. In cancer, hypoxia is associated with tumour progression and poor prognosis. Sustained hypoxia in growing tumours may lead to clinically aggressive phenotypes, increased invasive capacity, tumour cell metastasis, and resistance to both chemotherapy and radiation treatment [2, 3]. Oxygen tension in normal human tissues usually exceeds 40 mmHg; in contrast, oxygen tension in tumours may persist at 0–20 mmHg [4]. In normal cells, hypoxia usually induces growth arrest and causes death. However, under hypoxic conditions, tumour cells can adapt to poor nutrition and unfavourable microenvironments through genomic changes, thereby remaining vital [1]. In addition, cancer stem cells (CSC) are particularly responsible for hyper-adaptation to unfavorable TME. Indeed, CSC plays an important role in tumorigenesis and invasion/metastasis potential. Importantly, metabolic reprogramming is essential for maintaining the self-renewal of CSC [5, 6]. Studies also found that, as the tumour volume increases, the depletion of glucose will lead to the cytolysis and necrosis of tumour cells [7]. These suggests that metabolism may play an important role in tumorigenesis and development.

There are ten hallmarks including genome instability, inflammation, sustaining proliferative signaling, evading growth suppressors, resisting cell death, enabling replicative immortality, inducing angiogenesis, activating invasion and metastasis, reprogramming of energy metabolism and evading immune destruction in cancer [8]. As one of ten hallmarks in cancer, metabolic reprogramming has been extensively studied in the past two decades, and it has been widely accepted that carcinogenic transformation causes cancer cells to adapt to a well-defined metabolic phenotype, thereby profoundly affecting the tumour microenvironment (TME) [9]. Among these adaptations, reprogramming of glucose metabolism, one of the three major metabolic pathways, has been shown to be involved in mediating tumour growth [10]. Considering the effects of hypoxia and glucose metabolism on tumours, in this review, we summarize discoveries of hypoxia-related mechanisms that cause the metabolic reprogramming of human tumour cells.

## Metabolic adaptations to tumour cellular hypoxia

In general, oxygen and nutrient levels determine whether cells participate in mitochondrial respiration or glycolysis metabolism to balance the synthesis of ATP, macromolecules and reactive oxygen species (ROS). It is believed that the glycolysis efficiency of normal tissues is inhibited under normal oxygen; that is, they are characterized by the Pasteur effect. Glucose is mainly decomposed into pyruvate, which is then further decomposed by the mitochondrial tricarboxylic acid cycle and oxidative phosphorylation. In contrast, even under non-hypoxic conditions, malignant tumours exhibit a higher rate of glycolysis, a phenotype that allows carbon to be rapidly transferred from glycolysis into anabolic pathways at the expense of mitochondrial ATP synthesis [11]. This mandatory glycolysis phenotype was originally discovered by O. H. Warburg in dividing cancer cells; therefore, it is called the Warburg effect [12]. It has been suggested that the Warburg effect can induce cells to proliferate while preventing the production of ROS and oxidative stress, which are by-products of mitochondrial respiration [13]. From this perspective, enhanced glycolysis metabolism of tumour cells can both reduce oxidative stress and limit mitochondrial ATP synthesis. However, although the Warburg effect promotes the proliferation in a limited number of cell types under normoxic conditions, all human hypoxic tumour cells undergo glucose metabolism reprogramming regardless of their proliferation status [14]. Therefore, exploring the mechanism by which hypoxia regulates the adaptive switch of tumour cells to glucose metabolism may reveal new targets for use in tumour therapy.

## Cellular hypoxia adaptation is regulated by HIF

Several cellular mechanisms are involved in the adaptation to acute hypoxia, such as activation of ion channels through gas signalling in carotid body glomus cells and direct AMPK-induced upregulation of glycolysis in cardiomyocytes [15]. However, the main cellular response to hypoxia is mediated at the transcriptional level. Hypoxia activates a series of genes and microRNAs that maintain metabolic homeostasis that is regulated by HIF through transcriptional induction [16–18]. These genes facilitate the adaptation to decreasing O_2_ levels at the cell and organ levels. The continuous activation of hypoxia-inducible factor will destroy homeostasis, causing the body to be in a pathological state. The activation of HIF is regulated by a canonical pathway mediated by PHD, and the binding of some other proteins to HIF promote its stability.

### The canonical pathway of PHD-mediated regulation of HIF

Three members of the human HIF family have been identified: HIF-1, HIF-2, and HIF-3. These heterodimers are composed of α and β subunits, which dissociate under normal oxygen conditions [19]. HIF-1 and HIF-2 are the main transcription factors involved in cell adaptation to hypoxia [20]. HIF binds to the hypoxia response element (HRE) in the promoter region of the target and is involved in tumour cell survival, angiogenesis, glycolysis, and invasion/metastasis. HIF is a heterodimer consisting of a HIFα protein subunit expressed only during hypoxia and a constitutively expressed HIF-1β protein subunit. Under normoxic conditions, oxygen-dependent hydroxylation leads to the recognition of HIFα by the von Hippel-Lindau (pVHL) tumour suppressor, which recruits the E3 ubiquitin ligase, resulting in ubiquitination and protease degradation of HIFα [21, 22]. This prolyl-4-hydroxylase (PHD)-catalysed hydroxylation reaction is coupled with the oxidative decarboxylation of 2-oxoglutarate (2-OG), and succinate and carbon dioxide are produced [21]. Notably, all three PHD enzymes can utilize O_2_ as substrate and 2-OG, Fe^2+^ and ascorbic acid as co-substrates to hydroxylate both HIF-1α and HIF-2α. Compared to the loss of PDH2 heterozygosity or homozygous PDH3, a single lost PHD1 allele has the ability to induce hypoxia tolerance in mice, thus highlighting the functional specificity of PHD in vivo [23–25]. In vivo experiments, compared to the loss of heterozygous PDH2 or homozygous PDH3, a single lost mouse carrying PHD1 has the ability to induce hypoxia tolerance, thus highlighting the functional specificity of PHD in vivo [26]. Under hypoxia, the hydroxylation of HIFα is inhibited, leading to the stabilization of HIFα. HIFα dimerizes with HIF-1β to form a transcriptional activation complex. In addition, HIF asparaginyl hydroxylase or factor inhibiting HIF-1(FIH-1), a member of the Fe^2+^ and 2-OG-dependent dioxygenase family, can inhibit the transcriptional activity of HIFs by targeting the C-terminal transcription activation domain (CTAD) of HIF1-α and HIF-2α under normoxia to block the interaction between HIFα, p300 and CBP [27]. Importantly, due to the differences in the amino acid sequence of the protein subunits of the HIFα adjacent to the hydroxylated asparagine residue, the efficiency of CTAD hydroxylation of HIF-2α is lower than it is for HIF-1α [21, 28, 29]. Another difference is that HIF-1α expression is ubiquitous, while HIF-2α expression is restricted to specific tissues [30]. Furthermore, the heterogeneity of HIF protein isomers is also manifested by the lack of CTAD action with HIF-3α, which results in alternative splicing of HIF-3α to form an inhibitory PAS domain-containing protein, forming a transcriptionally inactive heterodimer with HIF-1α to inhibit the HIF reaction [19]. In addition to HIFα, FIH-1 has other substrates, the physiological functions of which need to be further explored [31, 32] (Fig. 1). In addition, some other potential targets of PHD, such as molecular scaffolds, may require structures to be effectively hydroxylated in tumour cells.

**Fig. 1:** Activation and degradation of HIFα. Under normoxic conditions, PHD uses 2-OG as a substrate and ascorbic acid and Fe^2+^ as co-substrates to catalyse the oxygen-dependent hydroxylation (OH) of HIFα (both HIF-1α and HIF-2α). Oxygen-dependent hydroxylation leads to the recognition of HIFα by the pVHL tumour suppressor, which recruits the E3 ubiquitin ligase, resulting in the ubiquitination and protease degradation of HIFα. Under hypoxia, the hydroxylation of HIFα is inhibited, leading to the stabilization of HIFα. HIFα dimerizes with HIF-1β to form a transcriptional activation complex, which binds to the HRE in the promoter region of target genes, inducing their transactivation

### Other proteins that promote the stability of HIF

PHD is known to promote the hydroxylation reaction of HIFα, thereby inducing the degradation of HIFα. Current research has revealed many proteins that can regulate the stability of HIF-1α. For example, overexpression of adenylate kinase 4 (AK4) promotes the stabilization of HIF-1α by increasing intracellular ROS levels, subsequently inducing the epithelial-mesenchymal transition (EMT) and enhancing tumour invasion potential under hypoxic conditions [33]; BRCA1-IRIS is a chromatin-associated replication and transcriptional regulator that is overexpressed in a variety of primary human cancers and can prevent glycogen synthase kinase-3 (GSK-3β) from recruiting F-box protein (Fbw7), a tumor suppressor associated with chromosomal instability and some types of malignancy, through phosphorylation of HIF. Fbw7 can further mediate ubiquitylation and degradation of HIF [34, 35]; Collagen prolyl 4-hydroxylase (P4H) is an essential catalytic enzyme in the progression of breast cancer. The α1 subunit of P4H (P4HA1) regulates the levels of 2-OG and succinic acid, suppressing the hydroxylation of proline in HIF-1α, thereby enhancing HIFα stability in cancer cells [36]. Additionally, HIF-induced proteins can also inhibit the degradation of HIFα through a feedback loop. The overexpression of HIF-2α in pancreatic cancer cells leads to the nuclear translocation of β-catenin, and the formation of the HIF-2α/β-catenin complex significantly prolongs the half-life of HIF-2α, maintaining the stability of HIF-2α [37]. These recently discovered proteins can be targeted to inhibit the stability of HIFα, thereby regulating tumor cell growth. Most of the proteins discovered in recent studies are described in detail in Table 1.

**Table 1:** Proteins that Promote the Stability of HIF

Cancer	Protein	Mechanism	Ref
liver, cervical	Bclaf1	Myb region of Bclaf1 participates in binding HIF-1α	[38]
lung	AK4	increase ROS levels	[33]
breast	HER2	/	[39]
liver	YAP	/	[40]
breast	FOXA1	/	[41]
breast	BRCA1-IRIS	prevents GSK-3β phosphorylation-driven degradation	[34]
breast	P4HA1	regulates the levels of 2-OG and succinic acid	[36]
myeloma	TRIM44	as a deubiquitinase of HIF-1α	[42]
colorectal	SOD3	decreases the activity of HIF-prolyl hydroxylase domain-containing protein	[43]
pancreatic	β-catenin	extends the half-life of HIF-2α	[37]
head and neck	GATA3	/	[44]

The importance of HIF in the microenvironment has made increasing researchers pay attention to the stability of HIF. However, current research has not fully explained the interaction mechanism between HIF and other molecules. For example, a recent study found that in hypoxic TME, enriched miR-301a-3p could be transmitted between GC cells via exosomes and then contributed to inhibit HIF-1α degradation through targeting PHD3 [45]. This means that extracellular vesicles (EVs) with proteins or RNA can regulate the stability of HIF in tumor cells. It has been widely recognized that HIF regulates the secretion of EVs under hypoxic conditions [46]. However, there are few studies on the negative feedback effect of EVs on the stability of HIF, which needs more in-depth research to explain the mechanism.

## Hypoxia regulates tumor glucose metabolism

The activation of HIF in a hypoxic environment can lead to the complex reprogramming of tumour cell glucose metabolism, summarized as follows: first, in terms of glucose catabolism, comprehensively enhanced glycolysis, glucose uptake and lactic acid formation regulate anaerobic oxidation and inhibit acetyl-CoA in the TCA cycle through pyruvate dehydrogenase (PDH) phosphorylation, which ultimately modulates aerobic oxidation; second, glycogen synthesis is regulated, and cancer cell glycogen reserves are increased; third, the bio-oxidation of glucose is increased by ROS production regulation, thereby inhibiting mitochondrial biogenesis and promoting mitochondrial clearance. The direct targets of HIFα and the HIFα-dependent genes that mediate these adaptations are illustrated in the metabolic pathway shown in Fig. 2.

**Fig. 2:** Hypoxic HIFα-Dependent Glucose Metabolic Reprogramming. Metabolic pathways illustrating HIFα transcriptional targets under hypoxia in tumor cells. Blue boxes, known HIFα targets. HIFα induces the expression of GLUT1, GLUT3, HK1/2 and LDHA, to increase glucose uptake and lactate formation. HIFα also induces the expression of PDK1, which then negatively regulates the entry of pyruvate to the TCA cycle. In addition, under hypoxic conditions, HIF-1 reduces the activity and respiration of complex I by inducing NDUFA4L2, and induces the expression of several microRNAs (miRNA) including miR-210, which can inhibit the assembly of ETC complex, thereby reducing the activity of ETC.

### HIF regulates glucose catabolism

Glucose catabolism mainly includes the anaerobic oxidation of sugar, aerobic oxidation of sugar and the pentose phosphate pathway, depending on the metabolic characteristics and oxygen supply status of different types of cells [47]. The Warburg effect allows tumour cells to gain survival advantages in two ways. One is to increase carbon sources, which are used to synthesize proteins, lipids, and nucleic acids to meet the needs of tumour growth; the other is to turn off aerobic oxidation channels to prevent the generation of free radicals, thereby preventing apoptosis [12]. Therefore, under hypoxic conditions, HIFα can regulate tumour growth by regulating the anaerobic and aerobic oxidation of glucose.

#### HIF regulates anaerobic glucose oxidation (glycolysis)

Current research has shown that hypoxia can regulate glucose anaerobic oxidation through the HIF-1α regulation of glucose transporters, glycolytic enzymes and NAD+, increasing glucose uptake and lactic acid formation, thereby promoting tumour growth. Tumour-associated macrophages (TAMs) induce increased expression of glucose transporters and glycolytic enzymes by stabilizing HIF-1α, including glucose transporter 1 (GLUT1), glucose transporter 3 (GLUT3), hexokinase-2 (HK2) and lactate dehydrogenase (LDH), to increase glucose uptake and lactate formation in breast cancer. The stabilizing effect of TAM on HIF-1α is achieved by an lncRNA (HISLA) in secreted EVs blocking the interaction between PDH2 and HIF-1α [48]. In addition to regulating the transcriptional activity of HIF-1α through PDH2, pyruvate kinase (PKM2) (whose mRNA is regulated by HIF-1α) can also act as a transcription coactivator, activating HIF-1α through feedback and inducing HIF-1α under hypoxic expression of glycolytic genes in HeLa cells [18, 49]. Subsequently, in non-small cell lung cancer, hypoxia-induced the lncRNA AC020978 can promote glycolysis metabolism by regulating the PKM2/HIF-1α axis [50]. Recently, it was also found that HIF-1α mediated protein kinase C(PKC)-induced upregulation of glycolytic genes, thereby promoting tumor cell proliferation in prostate cancer cells [51]. Another study of Tseng et al. revealed that transketolase (TKT), a metabolic enzyme involved in the non-oxidative branch of the pentose phosphate pathway (PPP), can increase the level of fumarate hydratase (FH) to promote the expression of HIF-1α, controlling breast cancer cell metastasis [52]. However, the promotion of HIF-1α on glycolysis will inevitably be negatively regulated. It has been confirmed that fructose-1,6-bisphosphatase (FBP1) can bind to the inhibitory domain of HIF-1α and restrict the growth of kidney cancer by inhibiting glycolysis [53].

In addition to glucose transporters and glycolytic enzymes, NAD+ also plays an irreplaceable role in the maintenance of glycolysis. In the presence of NADH, LDHA reduction of pyruvate to lactic acid is an important source of NAD+ regeneration. In hypoxic tumour cells, HIF-1α can induce the full expression of LDHA, which promotes the conversion of pyruvate to lactic acid and ensures the continuous production of NAD+ [14]. Interestingly, the level of nuclear NAD+ can also regulate the activity of HIF-1α. Lactic acid pretreatment can reduce the level of NAD+, thereby stabilizing HIF-1α and inducing a pseudohypoxic state, resulting in a decrease in the expression of the OXPHOS gene and reduction in ATP production [54].

#### HIF regulates aerobic glucose oxidation

Apart from the regulation of anaerobic oxidation, hypoxia induces LDHA and pyruvate dehydrogenase kinase 1 (PDK1) through HIF-1α to regulate pyruvate in the TCA cycle [54–56]. In cells with sufficient oxygen, pyruvate is transported to mitochondria and oxidized by pyruvate dehydrogenase (PDH) to acetyl-CoA, thus entering the TCA cycle. In contrast, under hypoxic conditions, on the one hand, HIF-1α induces the conversion of pyruvate to lactic acid, inhibiting its entry into the TCA cycle; on the other hand, HIF-1α induces the expression of pyruvate dehydrogenase kinase 1 (PDK1), followed by the phosphorylation of serine at PDK1-specific phosphorylation site 203 in PDH to inhibit PDH activity, resulting in a reduction in TCA cycle flux and limiting the production of mitochondrial NADH and FADH2 [55, 56]. Additionally, a recent study showed that HIF-1α can promote the expression of pyruvate dehydrogenase kinase 4(PDK4), further inducing macrophages polarize to M1 phenotype [57], which was described as a pro-inflammatory phenotype and tends to inhibit tumor progression [58]. Although this phenomenon occurs in carotid artery tissue, we can speculate that it may also occur in tumor cells. A decrease in reduction equivalents suppresses ETC, resulting in reduced electron transfer. Another important result of the decrease in TCA flux under hypoxia is a reduction in the production of aspartic acid, which is converted from oxaloacetic acid, a metabolite of the TCA cycle. Aspartic acid is necessary for nucleotide synthesis and cell proliferation. In a mouse model, cell hypoxia reduces aspartic acid levels, which in turn damages cell proliferation and tumour growth in vitro. In primary human tumours, aspartic acid levels are negatively correlated with hypoxic indicators [59]. Therefore, aspartic acid may be a metabolite that restricts tumour growth, and pathways related to the availability of aspartic acid may become targets for new cancer treatment.

In addition, the mitochondrial translocation of phosphoglycerate kinase 1 (PGK1) can also act as a protein kinase to activate PDK1 and inhibit the activity of PDH, thereby inhibiting the TCA cycle and eventually leading to the occurrence of brain tumours. Under hypoxia, HIF-1α induces the binding of PGK1 to the mitochondrial outer membrane translocation enzyme (TOM) complex and enters the mitochondria; in addition, HIF-1α promotes the binding of PIN1 and PGK1, thereby regulating the binding of PGK1 and TOM [60].

### HIF regulates glycogen metabolism

In addition to regulating glucose catabolism, HIF can increase cancer glycogen reserves [61] under hypoxia. Pelletier et al. found that the glycogen content of cancer cell lines cultured in 1% oxygen increased from 5 to 37-fold, indicating that the synthesis of glycogen is HIF-1α-dependent. Within 24 h of glucose removal from the culture medium, cells that accumulate glycogen under hypoxic conditions have higher viability (70–80%) than cells cultured under normoxic conditions (20–60%) [62]. In addition, PHD2 gene inactivation or systemic pharmacological inhibition in neutrophils can lead to the stabilization of non-hypoxic HIF-1α, thereby enhancing glycogen storage. Therefore, it is necessary to understand how HIF regulates glycogen metabolism. Glycogen originates from the allosteric formation of glucose-6-phosphate (G6P), glucose-1-phosphate (G1P) and uridine triphosphate (UTP) to form uridine diphosphate glucose (UDPG) [61]. UDPG is connected by α-1,4-glycosidic bonds to form a straight chain and connected by α-1,6-glycosidic bonds to form branches, and these formed branches can increase the water solubility of glycogen.

The synthesis and decomposition of glycogen involve the activities of various enzymes and regulatory proteins. Among these, glycogen synthase (GS) and glycogen phosphorylase (GP) are key enzymes in the process of catalysing glycogen synthesis and degradation, respectively. GS elongates the glycogen branch by forming an α-1,4 glycosidic bridge, while GP cleaves these glycogens, releasing G1P, which enters the glycolysis pathway, or G6P that enters the PPP [63]. This result suggests that the pathways by which HIF regulates glycogen metabolism include the key regulatory enzymes and related kinases of glycogen synthesis and decomposition. Studies have shown that under hypoxic conditions, HIF not only upregulates the expression of UDP-glucose pyrophosphorylase and promotes glucose activation before glycogen synthesis but also inhibits liver glycogen phosphorylase (PYGL) by promoting glycogen synthase 1 (GYS1) regulation of glycogen synthesis. Moreover, the activation of glycogen branching enzyme (GBE1) by HIF can further regulate the formation of glycogen branches [56, 63]. Interestingly, direct regulation of key enzymes is not the only mechanism by which glycogen metabolism is modulated. In fact, indirect effects on key enzymes can also regulate glycogen synthesis. For example, the HIF-1α-dependent expression of PP1 complex phosphatase (PPP1R3C) in human MCF7 cells activates GYS1 while reducing the breakdown of glycogen into glucose monomers [64]. These HIF-dependent effects allow glycogen to accumulate under conditions of hypoxia and nutritional deficiencies, affecting cell responses.

### HIF regulates the biological oxidation of glucose

Mitochondria, organelles that generate energy in the body, are composed of simple organophospholipid bilayer membranes, intermembrane spaces, complex internal phospholipid bilayers, and mitochondrial matrices. They are especially enriched in the heart muscle, skeletal muscle, liver, kidney, and especially neuronal cells, which need high levels of energy to function [65]. The biological oxidation of glucose is a precise process that relies on the oxidized the mitochondrial respiratory chain to transfer electrons from NADH and succinate to oxygen and finally the combination of hydrogen protons and oxygen to form water and release ATP [66]. The oxidized respiratory chain consists of four mitochondrial complexes located on the inner mitochondrial membrane, called complexes I, II, III, and IV. They are NADH-CoQ reductase, succinate-CoQ reductase, CoQ-cytochrome c reductase, and cytochrome c oxidase. Ubiquinone (CoQ) and cytochrome c are two freely diffusible molecules that mediate electron transfer between complexes [67]. Current research shows that HIF can regulate the biological oxidation of glucose through the regulation of mitochondria in a hypoxic environment, including the regulation of mitochondrial biogenesis, the generation of ROS [68, 69] and the removal of mitochondria.

#### HIF inhibits mitochondrial biogenesis

Because of the important role of mitochondria in energy production, the regulation of mitochondrial biogenesis by HIF under hypoxia is an important mechanism by which biological oxidation is regulated. According to reports, in kidney cancer cells lacking VHL, HIF-1α can negatively regulate mitochondrial mass and O_2_ consumption. Further in vitro experiments showed that Myc-transformed cancer cells exhibited an increased mitochondrial mass and increased rate of oxygen consumption. Furthermore, it has been reported that Myc-overexpressing tumor cells are exquisitely sensitive to the inhibitor of the mitochondrial electron transport chain. Myc-induced transformation from oxidation glucose as the main strategy to the conversion essential to the activity substrate. This paradoxical phenomenon can be explained by the accumulation of glutamine, the major catabolizing bio-energetic substrates in mitochondrial TCA cycle. Myc-induced transformation leads to the conversion from glucose to glutamine as the oxidizable substrate which is essential to maintain TCA cycle activity [70]. HIF-1α not only can bind and activate the transcription of the MXI-1 gene, thereby inhibiting the transcriptional activity of c-Myc through its encoded product but can also promote the degradation of c-Myc in an independent manner through MXI-1. More specifically, c-Myc regulates mitochondrial biogenesis by inhibiting PGC-1β [56, 71, 72]. In a recent study, researchers established transgenic mice with liver-specific PGC-1β overexpression (LivPGC-1β) and PGC-1β gene knockout (LivPGC-1βKO), and in vivo experiments demonstrated that PGC-1β played a key role in driving tumour development [73]. In addition, the role of PGC-1α in promoting mitochondrial biogenesis was also confirmed in a recent study [74] but did not confirm whether it was also targeted by HIF in tumour cells. Additionally, HIF-1α can inhibit mitochondrial biogenesis by inhibiting the expression of PINK1, an essential gene for mitochondrial biogenesis. The HEY1 gene is an important member of the HEY family, which mainly functions to recruit corepressors for its target genes to inhibit transcription. Under hypoxia, HIF-1α can upregulate the expression of HEY1 and then recruit corepressors to inhibit the transcriptional activity of PINK1, reducing mitochondrial mass and promoting the growth of cancer cells [75]. In summary, the inhibition of mitochondrial biogenesis by HIF depends mainly on the regulation of key genes, such as c-Myc, PGC-1, and PINK1, which may also provide new therapeutic targets for future cancer treatment. However, it is not unclear that the mechanisms underlying how hypoxia is sensed to trigger mitophagy.

#### HIF regulates mitochondrial ROS production

When the balance between the production and utilization of oxidant molecules is disrupted, oxidative stress occurs. As observed in an ischaemia/reperfusion model, excessive production of ROS during oxidative stress may cause protein, DNA, and lipid damage, thereby causing cell damage [76, 77]. Active oxygen includes hydrogen peroxide, hydroxyl radicals and superoxide anions, which are mainly produced in complexes I and III of the mitochondrial inner membrane [78–82] (Fig. 3). Moreover, other sources of ROS, including lipoxygenase, peroxisomes and NADPH oxidase, can also regulate the production of ROS [83–85]. In healthy individuals, hypoxia increases mitochondrial ROS to induce HIF-dependent induction of human telomerase [G] (hTERT) gene expression to extend the cell lifespan, while hypoxia increases the activity of complexes I and III in tumour cells, limiting the production of ROS, preventing tumour cells from being damaged, and promoting tumour growth [86–88].

**Fig. 3:** Sites where hypoxia inhibits ROS production. Hypoxia increases the activity of complexes I and III in tumour cells, limiting the production of ROS. NADPH oxidase can also regulate the production of ROS, which may become a potential site regulated by HIFα

A recent study showed that NADH dehydrogenase (ubiquinone) 1 alpha subcomplex 4-like 2 (NDUFA4L2) is highly overexpressed in hypoxic liver cancer cells, and it has been confirmed that NDUFA4L2 is regulated by HIF-1α in HCC cells. Inactivation of HIF-1α/NDUFA4L2 increased mitochondrial activity and oxygen consumption, resulting in ROS accumulation and apoptosis, which further inhibited the growth and spread of HCC [89]. Coincidentally, the effect of HIF/NDUFA4L2 on ROS production is also found in kidney cancer [90] and lung cancer [91], suggesting the universal applicability of this signalling pathway in cancer cells. Further research found that NDUFA4L2 appears to affect ETC activity by specifically inhibiting complex I [69]. As an important part of protease complex I, Fe-S clusters participate in electron transport and oxidative phosphorylation [92]. Notably, the biogenesis of Fe-S clusters depends on the assembly protein ISCU1/2 [93]. Therefore, once the expression of ISCU1/2 is inhibited, the activity of complex I is inhibited. Researchers have found that the expression of miR-210 is significantly increased by the transcriptional activation of HIFα in vitro in kidney cancer tissues under hypoxic conditions [94]. Importantly, miR-210 can significantly inhibit ISCU1/2 protein expression, resulting in the destruction of iron-sulfur cluster integrity and limiting ROS production [94, 95].

In addition, complex III can also participate in the process of hypoxic ROS production. After RNAi interferes with Rieske iron-sulfur protein (RISP) in complex III, hypoxia-induced HIF-1α stabilization is attenuated, and ROS production is decreased, suggesting a strong link between ROS production and complex III and HIF-1α stabilization [68]. Moreover, in HeLa cells, HIF-1α induces the transcription of genes encoding COX4-i2 and LON, a mitochondrial protease that is required for COX4-i1 degradation [96]. Although its role in tumour cells has not been confirmed, COX4-i2 can increase the production of ROS in hypoxic carotid body spherical cells [97], suggesting that COX4i2 may play the same function in tumour cells. Additionally, more recently, the emerging concept of the “reverse Warburg effect”, involving the regulation of energy metabolism by ROS, has attracted considerable attention. Tumor cell derived ROS decrease the expression of caveolin-1 in cancer-associated fibroblasts (CAFs). Loss of caveolin-1 in CAFs also results in elevated ROS levels, which in turn stabilize HIF-1α [98, 99].

In summary, under hypoxic conditions, HIF mainly regulates the activity of mitochondrial complexes to induce the production of ROS, which may become a potential strategy for the treatment of cancer.

#### HIF promotes mitochondrial clearance

In addition to inhibiting the production of mitochondria, HIF can also reduce the mass of mitochondria by promoting mitochondrial clearance. Current research shows that HIF-1α promotes mitochondrial clearance in tumour cells mainly by inducing mitochondrial autophagy, also referred as mitophagy [100]. Mechanically, mitophagy serves as an adaptive metabolic response that prevents accumulation of high levels of ROS by removing old/damaged mitochondria. Mitochondrial permeability transition is thought to be responsible for the mitophagy of depolarized mitochondria, there by generating cytotoxic ROS [101]. Further research showed that HIF-1α upregulates BNIP3 expression under hypoxic conditions, thereby inducing Beclin1-dependent mitophagy and mitochondrial metabolic reprogramming, resulting in reduced ROS production and promoted tumour growth [102, 103]. Furthermore, BNIP3-dependent mitochondrial autophagy leads to enhanced RGC neuroglycolysis, which in turn promotes the differentiation of macrophages into the M1 phenotype during inflammation [104]. Therefore, the regulation of the inflammatory response by BNIP3-dependent mitophagy may also be another possible mechanism that has not been proven to affect tumorigenesis and development.

## Therapeutic strategy by targeting HIF in Cancer metabolism

Since HIF can regulate the energy metabolism of cancer cells through multiple channels under hypoxic conditions and promote the survival of cancer cells, inhibiting the cancer metabolism pathway mediated by HIF or HIF may become one of the potential treatment methods for cancer [105–107]. It has been discovered that many drugs, such as aspirin [108] and Tamoxifen [109], can block the growth of tumors by inhibiting the expression or activity of HIF-1α thereby providing new anti-cancer treatments. On the other hand, drugs targeting HIF-1α mediated metabolic enzymes may also affect tumor cell proliferation induced by hypoxia. For example, the inhibition of Metformin on PDH [110], Cetuximab on LDHA [111] and Dovitinib on GLUT [112] expression will change the ability of cancer cells to metabolize pyruvate to lactic acid, leading to a decline in tumor growth. The above examples also remind us that drug-repositioning (DR), an attractive approach that can facilitate the drug discovery process by repurposing existing pharmaceuticals to treat illnesses other than their primary indications, may be a promising therapeutic strategy, such as metformin that is a traditional medicine for treating diabetes [113]. Moreover, the enhanced glucose metabolism induced by HIF-1α can also lead to the resistance of Gemcitabine to pancreatic cancer [114]. However, the role of HIF and HIF-regulated metabolic enzymes in tumor resistance is still unclear, and further research is needed.

Metabolic reprogramming in cancer cells induced by hypoxia is a complex event that cannot be simply explained as the transition from OXPHOS to aerobic glycolysis.

The development of drugs targeting HIF or HIF mediated metabolic enzymes will become a new potential method for the treatment of cancer (Table 2).

**Table 2:** Drugs targeting HIF/HIF mediated metabolic enzymes

Drug	Target	Tumor	Ref
Atorvastatin	HIF-1α	Burkitt’s Lymphoma	[115]
Oxaliplatin	HIF-1α	Colorectal cancer	[116]
Tamoxifen	HIF-1α	Breast cancer	[109]
Trichostatin A	HIF-1α	Cervical cancer	[117]
Diacetoxyscirpenol	HIF-1α	Liver cancer	[118]
Metformin	HIF-1α	Breast cancer	[119]
Metformin	HIF-1α/GLUT, HK2, PKM, LDH	Cervical cancer	[120]
Ginsenoside Compound K	HIF-1α/PDK1	Lung cancer	[121]
Dovitinib	HIF-1α/GLUT	Lung cancer	[112]
Metformin	HIF-1α/PDH	Oral cancer	[110]
Cetuximab	HIF-1α/LDHA	Head and neck cancer	[111]
Troxacitabine	HIF-1α/PGK	Lung cancer	[122]

## Conclusion

The remarkable metabolic adaptability of hypoxic human tumour cells can be understood as a balance among energy production, sufficient macromolecule biosynthesis and redox balance preservation of tumour cells. The process of metabolic adaptation must be studied in depth to determine the weakness of tumour metabolic pathways and to formulate an effective treatment strategy. Since the early nineteenth century, scientists have discovered a fascinating new level of complexity that has added to our understanding of molecular and cellular mechanisms, onto which is superimposed the biochemical metabolic network that has been recently dissected and characterized. This wealth of knowledge illustrates that HIF regulates the adaptation of tumour cells to undertake glucose metabolism through the regulation of glucose anaerobic oxidation, aerobic oxidation, glycogen and biological oxidation. Clarifying the molecular mechanism of HIF-mediated hypoxia driving metabolic changes at the cellular level will help to strategically focus on certain pathways for designing improved therapeutic strategies to treat cancers.

## Data Availability

The datasets are available from the corresponding author on reasonable request.

## Abbreviations

A-CoA: Acetyl-Coenzyme-A
AK4: Adenylate kinase 4
BNIP3: BCL2/adenovirus E1B-19 kDa interacting protein 3
BNIP3L: BCL2/adenovirus E1B-19 kDa interacting protein 3-like
1,3BPG: 1,3 diphosphoglycerate
3-PGA: 3-phosphoglycerate
CAFs: Cancer-associated fibroblasts
CSC: Cancer stem cells
COX4-i1/2: Cytochrome c oxidase subunit 4, isoform 1/2
DR: Drug-repositioning
EMT: Epithelial-mesenchymal transition
EVs: Extracellular vesicles
FBP1: Fructose-1,6-bisphosphatase
Fbw7: F-box protein
FH: Fumarate hydratase
FOXA1: Foxhead box A1
GATA3: GATA binding protein 3
GBE1: 1,4a-glucan branching enzyme
GLUT1/3: Glucose transporter 1/3 (encoded by Slc2a1 and Slc2a3, respectively)
GSK-3β: Glycogen synthase kinase-3
G1P: Glucose-1-phosphatase
G6P: Glucose-6-phosphatase
GYS1: Glycogen synthase
HER2: Human Epidermal Growth Factor Receptor 2
HK1/2: Hexokinase 1/2
HIF: Hypoxia-inducible Factor
ISCU1/2: Iron–sulfur cluster assembly enzyme 1/2
LDHA: Lactate dehydrogenase A
MAX: Myc-associated factor
MXI1: MAX interactor 1
NDUFA4L2: NADH dehydrogenase (ubiquinone) 1a subcomplex subunit 4-like 2
NHE1: Na+/K+ exchanger 1
2-OG: 2-oxoglutarate
PDH: Pyruvate dehydrogenase
PDK1: Pyruvate dehydrogenase kinase 1
PKC: Protein kinase C
P4H: Collagen prolyl 4-hydroxylase
P4HA1: α1 subunit of P4H
PGC1b: PPARg coactivator 1b
PGK1: Phosphoglycerate kinase 1
PGM1: Phosphoglucomutase 1
PKM: Pyruvate kinase, muscle (includes PKM1 and M2)
PPP1R3C: Protein phosphatase 1 regulatory subunit 3C
PYGL: Glycogen phosphorylase, liver
ROS: Reactive oxygen species
SOD3: Superoxide dismutase
TAM: Tumour-associated macrophage
TKT: Transketolase
TRIM44: Tripartite motif containing 44
UDPG: UDP-glucose
Ub: Ubiquitination
YAP: Yes-associated Protein

## References

[1] Vaupel P, Harrison L (2004). Tumor hypoxia: causative factors, compensatory mechanisms, and cellular response. Oncologist.

[2] Hockel M, Vaupel P (2001). Tumor hypoxia: definitions and current clinical, biologic, and molecular aspects. J Natl Cancer Inst.

[3] Muz B, de la Puente P, Azab F, Azab AK (2015). The role of hypoxia in cancer progression, angiogenesis, metastasis, and resistance to therapy. Hypoxia (Auckl).

[4] Vaupel P, Kallinowski F, Okunieff P (1989). Blood flow, oxygen and nutrient supply, and metabolic microenvironment of human tumors: a review. Cancer Res.

[5] Yoshida GJ (2015). Metabolic reprogramming: the emerging concept and associated therapeutic strategies. J Exp Clin Cancer Res.

[6] Yoshida GJ, Saya H (2016). Therapeutic strategies targeting cancer stem cells. Cancer Sci.

[7] Vaupel P (1977). Hypoxia in neoplastic tissue. Microvasc Res.

[8] Hanahan D, Weinberg RA (2011). Hallmarks of cancer: the next generation. Cell.

[9] Bader JE, Voss K, Rathmell JC (2020). Targeting metabolism to improve the tumor microenvironment for Cancer immunotherapy. Mol Cell.

[10] Tsegaye MA, Schafer ZT (2017). Collapsing the metabolic PON2zi scheme in pancreatic ductal adenocarcinoma. Trends Cell Biol.

[11] Vander Heiden MG, Cantley LC, Thompson CB (2009). Understanding the Warburg effect: the metabolic requirements of cell proliferation. Science.

[12] Warburg O (1956). On the origin of cancer cells. Science.

[13] Gruning NM, Rinnerthaler M, Bluemlein K, Mulleder M, Wamelink MM, Lehrach H, Jakobs C, Breitenbach M, Ralser M (2011). Pyruvate kinase triggers a metabolic feedback loop that controls redox metabolism in respiring cells. Cell Metab.

[14] Schito L, Rey S (2018). Cell-autonomous metabolic reprogramming in hypoxia. Trends Cell Biol.

[15] Bargiela D, Burr SP, Chinnery PF (2018). Mitochondria and hypoxia: metabolic crosstalk in cell-fate decisions. Trends Endocrinol Metab.

[16] Ivan M, Kaelin WG (2017). The EGLN-HIF O2-sensing system: multiple inputs and feedbacks. Mol Cell.

[17] Schito L, Semenza GL (2016). Hypoxia-inducible factors: master regulators of Cancer progression. Trends Cancer.

[18] Semenza GL, Roth PH, Fang HM, Wang GL (1994). Transcriptional regulation of genes encoding glycolytic enzymes by hypoxia-inducible factor 1. J Biol Chem.

[19] Weidemann A, Johnson RS (2008). Biology of HIF-1alpha. Cell Death Differ.

[20] Keith B, Johnson RS, Simon MC (2011). HIF1alpha and HIF2alpha: sibling rivalry in hypoxic tumour growth and progression. Nat Rev Cancer.

[21] Kaelin WG, Ratcliffe PJ (2008). Oxygen sensing by metazoans: the central role of the HIF hydroxylase pathway. Mol Cell.

[22] Semenza GL (2012). Hypoxia-inducible factors in physiology and medicine. Cell.

[23] Bruick RK, McKnight SL (2001). A conserved family of prolyl-4-hydroxylases that modify HIF. Science.

[24] Epstein AC, Gleadle JM, McNeill LA, Hewitson KS, O'Rourke J, Mole DR, Mukherji M, Metzen E, Wilson MI, Dhanda A, Tian YM, Masson N, Hamilton DL, Jaakkola P, Barstead R, Hodgkin J, Maxwell PH, Pugh CW, Schofield CJ, Ratcliffe PJ (2001). C. elegans EGL-9 and mammalian homologs define a family of dioxygenases that regulate HIF by prolyl hydroxylation. Cell.

[25] Markolovic S, Wilkins SE, Schofield CJ (2015). Protein hydroxylation catalyzed by 2-Oxoglutarate-dependent Oxygenases. J Biol Chem.

[26] Aragones J, Schneider M, Van Geyte K, Fraisl P, Dresselaers T, Mazzone M, Dirkx R, Zacchigna S, Lemieux H, Jeoung NH, Lambrechts D, Bishop T, Lafuste P, Diez-Juan A, Harten SK, Van Noten P, De Bock K, Willam C, Tjwa M, Grosfeld A, Navet R, Moons L, Vandendriessche T, Deroose C, Wijeyekoon B, Nuyts J, Jordan B, Silasi-Mansat R, Lupu F, Dewerchin M, Pugh C, Salmon P, Mortelmans L, Gallez B, Gorus F, Buyse J, Sluse F, Harris RA, Gnaiger E, Hespel P, Van Hecke P, Schuit F, Van Veldhoven P, Ratcliffe P, Baes M, Maxwell P, Carmeliet P (2008). Deficiency or inhibition of oxygen sensor Phd1 induces hypoxia tolerance by reprogramming basal metabolism. Nat Genet.

[27] Lee P, Chandel NS, Simon MC (2020). Cellular adaptation to hypoxia through hypoxia inducible factors and beyond. Nat Rev Mol Cell Biol.

[28] Bracken CP, Fedele AO, Linke S, Balrak W, Lisy K, Whitelaw ML, Peet DJ (2006). Cell-specific regulation of hypoxia-inducible factor (HIF)-1alpha and HIF-2alpha stabilization and transactivation in a graded oxygen environment. J Biol Chem.

[29] Schito L, Rey S (2017). Hypoxic pathobiology of breast cancer metastasis. Biochim Biophys Acta Rev Cancer.

[30] Hu CJ, Wang LY, Chodosh LA, Keith B, Simon MC (2003). Differential roles of hypoxia-inducible factor 1alpha (HIF-1alpha) and HIF-2alpha in hypoxic gene regulation. Mol Cell Biol.

[31] Cockman ME, Webb JD, Kramer HB, Kessler BM, Ratcliffe PJ (2009). Proteomics-based identification of novel factor inhibiting hypoxia-inducible factor (FIH) substrates indicates widespread asparaginyl hydroxylation of ankyrin repeat domain-containing proteins. Mol Cell Proteomics.

[32] Zhang N, Fu Z, Linke S, Chicher J, Gorman JJ, Visk D, Haddad GG, Poellinger L, Peet DJ, Powell F, Johnson RS (2010). The asparaginyl hydroxylase factor inhibiting HIF-1alpha is an essential regulator of metabolism. Cell Metab.

[33] Jan YH, Lai TC, Yang CJ, Lin YF, Huang MS, Hsiao M (2019). Adenylate kinase 4 modulates oxidative stress and stabilizes HIF-1alpha to drive lung adenocarcinoma metastasis. J Hematol Oncol.

[34] Li AG, Murphy EC, Culhane AC, Powell E, Wang H, Bronson RT, Von T, Giobbie-Hurder A, Gelman RS, Briggs KJ, Piwnica-Worms H, Zhao JJ, Kung AL, Kaelin WG, Livingston DM (2018). BRCA1-IRIS promotes human tumor progression through PTEN blockade and HIF-1alpha activation. Proc Natl Acad Sci U S A.

[35] Flugel D, Gorlach A, Kietzmann T (2012). GSK-3beta regulates cell growth, migration, and angiogenesis via Fbw7 and USP28-dependent degradation of HIF-1alpha. Blood.

[36] Xiong G, Stewart RL, Chen J, Gao T, Scott TL, Samayoa LM, O'Connor K, Lane AN, Xu R (2018). Collagen prolyl 4-hydroxylase 1 is essential for HIF-1alpha stabilization and TNBC chemoresistance. Nat Commun.

[37] Zhang Q, Lou Y, Zhang J, Fu Q, Wei T, Sun X, Chen Q, Yang J, Bai X, Liang T (2017). Hypoxia-inducible factor-2alpha promotes tumor progression and has crosstalk with Wnt/beta-catenin signaling in pancreatic cancer. Mol Cancer.

[38] Shao A, Lang Y, Wang M, Qin C, Kuang Y, Mei Y, Lin D, Zhang S, Tang J (2020). Bclaf1 is a direct target of HIF-1 and critically regulates the stability of HIF-1alpha under hypoxia. Oncogene.

[39] Jarman EJ, Ward C, Turnbull AK, Martinez-Perez C, Meehan J, Xintaropoulou C, Sims AH, Langdon SP (2019). HER2 regulates HIF-2alpha and drives an increased hypoxic response in breast cancer. Breast Cancer Res.

[40] Zhang X, Li Y, Ma Y, Yang L, Wang T, Meng X, Zong Z, Sun X, Hua X, Li H (2018). Yes-associated protein (YAP) binds to HIF-1alpha and sustains HIF-1alpha protein stability to promote hepatocellular carcinoma cell glycolysis under hypoxic stress. J Exp Clin Cancer Res.

[41] Fu X, Pereira R, De Angelis C, et al. FOXA1 upregulation promotes enhancer and transcriptional reprogramming in endocrine-resistant breast cancer. Proc Natl Acad Sci U S A. 2019;116(52):26823–34.10.1073/pnas.1911584116PMC693643631826955

[42] Chen Z, Lin TC, Bi X, Lu G, Dawson BC, Miranda R, Medeiros LJ, McNiece I, McCarty N (2019). TRIM44 promotes quiescent multiple myeloma cell occupancy and survival in the osteoblastic niche via HIF-1alpha stabilization. Leukemia.

[43] Mira E, Carmona-Rodriguez L, Perez-Villamil B, Casas J, Fernandez-Acenero MJ, Martinez-Rey D, Martin-Gonzalez P, Heras-Murillo I, Paz-Cabezas M, Tardaguila M, Oury TD, Martin-Puig S, Lacalle RA, Fabrias G, Diaz-Rubio E, Manes S (2018). SOD3 improves the tumor response to chemotherapy by stabilizing endothelial HIF-2alpha. Nat Commun.

[44] Lin MC, Lin JJ, Hsu CL, Juan HF, Lou PJ, Huang MC (2017). GATA3 interacts with and stabilizes HIF-1alpha to enhance cancer cell invasiveness. Oncogene.

[45] Xia X, Wang S, Ni B, et al. Hypoxic gastric cancer-derived exosomes promote progression and metastasis via MiR-301a-3p/PHD3/HIF-1α positive feedback loop. Oncogene. 2020. 10.1038/s41388-020-01425-6.10.1038/s41388-020-01425-632826951

[46] Peng X, Yang L, Ma Y, Li Y, Li H (2020). Focus on the morphogenesis, fate and the role in tumor progression of multivesicular bodies. Cell Commun Signal.

[47] Li Z, Zhang H (2016). Reprogramming of glucose, fatty acid and amino acid metabolism for cancer progression. Cell Mol Life Sci.

[48] Chen F, Chen J, Yang L, Liu J, Zhang X, Zhang Y, Tu Q, Yin D, Lin D, Wong PP, Huang D, Xing Y, Zhao J, Li M, Liu Q, Su F, Su S, Song E (2019). Extracellular vesicle-packaged HIF-1alpha-stabilizing lncRNA from tumour-associated macrophages regulates aerobic glycolysis of breast cancer cells. Nat Cell Biol.

[49] Luo W, Hu H, Chang R, Zhong J, Knabel M, O'Meally R, Cole RN, Pandey A, Semenza GL (2011). Pyruvate kinase M2 is a PHD3-stimulated coactivator for hypoxia-inducible factor 1. Cell.

[50] Hua Q, Mi B, Xu F, Wen J, Zhao L, Liu J, Huang G (2020). Hypoxia-induced lncRNA-AC020978 promotes proliferation and glycolytic metabolism of non-small cell lung cancer by regulating PKM2/HIF-1alpha axis. Theranostics.

[51] Xu W, Zeng F, Li S, Li G, Lai X, Wang QJ, Deng F (2018). Crosstalk of protein kinase C epsilon with Smad2/3 promotes tumor cell proliferation in prostate cancer cells by enhancing aerobic glycolysis. Cell Mol Life Sci.

[52] Tseng CW, Kuo WH, Chan SH, Chan HL, Chang KJ, Wang LH (2018). Transketolase regulates the metabolic switch to control breast Cancer cell metastasis via the alpha-Ketoglutarate signaling pathway. Cancer Res.

[53] Li B, Qiu B, Lee DS, Walton ZE, Ochocki JD, Mathew LK, Mancuso A, Gade TP, Keith B, Nissim I, Simon MC (2014). Fructose-1,6-bisphosphatase opposes renal carcinoma progression. Nature.

[54] Gomes AP, Price NL, Ling AJ, Moslehi JJ, Montgomery MK, Rajman L, White JP, Teodoro JS, Wrann CD, Hubbard BP, Mercken EM, Palmeira CM, de Cabo R, Rolo AP, Turner N, Bell EL, Sinclair DA (2013). Declining NAD(+) induces a pseudohypoxic state disrupting nuclear-mitochondrial communication during aging. Cell.

[55] Dupuy F, Tabaries S, Andrzejewski S, Dong Z, Blagih J, Annis MG, Omeroglu A, Gao D, Leung S, Amir E, Clemons M, Aguilar-Mahecha A, Basik M, Vincent EE, St-Pierre J, Jones RG, Siegel PM (2015). PDK1-dependent metabolic reprogramming dictates metastatic potential in breast Cancer. Cell Metab.

[56] Semenza GL (2013). HIF-1 mediates metabolic responses to intratumoral hypoxia and oncogenic mutations. J Clin Invest.

[57] Han X, Ma W, Zhu Y, Sun X, Liu N (2020). Advanced glycation end products enhance macrophage polarization to the M1 phenotype via the HIF-1alpha/PDK4 pathway. Mol Cell Endocrinol.

[58] Sica A, Bronte V (2007). Altered macrophage differentiation and immune dysfunction in tumor development. J Clin Invest.

[59] Garcia-Bermudez J, Baudrier L, La K, Zhu XG, Fidelin J, Sviderskiy VO, Papagiannakopoulos T, Molina H, Snuderl M, Lewis CA, Possemato RL, Birsoy K (2018). Aspartate is a limiting metabolite for cancer cell proliferation under hypoxia and in tumours. Nat Cell Biol.

[60] Li X, Jiang Y, Meisenhelder J, Yang W, Hawke DH, Zheng Y, Xia Y, Aldape K, He J, Hunter T, Wang L, Lu Z (2016). Mitochondria-Translocated PGK1 functions as a protein kinase to coordinate glycolysis and the TCA cycle in tumorigenesis. Mol Cell.

[61] Dauer P, Lengyel E (2019). New roles for glycogen in tumor progression. Trends Cancer.

[62] Pelletier J, Bellot G, Gounon P, Lacas-Gervais S, Pouyssegur J, Mazure NM (2012). Glycogen synthesis is induced in hypoxia by the hypoxia-inducible factor and promotes Cancer cell survival. Front Oncol.

[63] Favaro E, Bensaad K, Chong MG, Tennant DA, Ferguson DJ, Snell C, Steers G, Turley H, Li JL, Gunther UL, Buffa FM, McIntyre A, Harris AL (2012). Glucose utilization via glycogen phosphorylase sustains proliferation and prevents premature senescence in cancer cells. Cell Metab.

[64] Shen GM, Zhang FL, Liu XL, Zhang JW (2010). Hypoxia-inducible factor 1-mediated regulation of PPP1R3C promotes glycogen accumulation in human MCF-7 cells under hypoxia. FEBS Lett.

[65] Palade GE (1953). An electron microscope study of the mitochondrial structure. J Histochem Cytochem.

[66] Sun F, Zhou Q, Pang X, Xu Y, Rao Z (2013). Revealing various coupling of electron transfer and proton pumping in mitochondrial respiratory chain. Curr Opin Struct Biol.

[67] Ham PB, Raju R (2017). Mitochondrial function in hypoxic ischemic injury and influence of aging. Prog Neurobiol.

[68] Guzy RD, Hoyos B, Robin E, Chen H, Liu L, Mansfield KD, Simon MC, Hammerling U, Schumacker PT (2005). Mitochondrial complex III is required for hypoxia-induced ROS production and cellular oxygen sensing. Cell Metab.

[69] Tello D, Balsa E, Acosta-Iborra B, Fuertes-Yebra E, Elorza A, Ordonez A, Corral-Escariz M, Soro I, Lopez-Bernardo E, Perales-Clemente E, Martinez-Ruiz A, Enriquez JA, Aragones J, Cadenas S, Landazuri MO (2011). Induction of the mitochondrial NDUFA4L2 protein by HIF-1alpha decreases oxygen consumption by inhibiting complex I activity. Cell Metab.

[70] Yoshida GJ (2018). Emerging roles of Myc in stem cell biology and novel tumor therapies. J Exp Clin Cancer Res.

[71] Li F, Wang Y, Zeller KI, Potter JJ, Wonsey DR, O'Donnell KA, Kim JW, Yustein JT, Lee LA, Dang CV (2005). Myc stimulates nuclearly encoded mitochondrial genes and mitochondrial biogenesis. Mol Cell Biol.

[72] Zhang H, Gao P, Fukuda R, Kumar G, Krishnamachary B, Zeller KI, Dang CV, Semenza GL (2007). HIF-1 inhibits mitochondrial biogenesis and cellular respiration in VHL-deficient renal cell carcinoma by repression of C-MYC activity. Cancer Cell.

[73] Piccinin E, Peres C, Bellafante E, Ducheix S, Pinto C, Villani G, Moschetta A (2018). Hepatic peroxisome proliferator-activated receptor gamma coactivator 1beta drives mitochondrial and anabolic signatures that contribute to hepatocellular carcinoma progression in mice. Hepatology.

[74] Cox CS, McKay SE, Holmbeck MA, Christian BE, Scortea AC, Tsay AJ, Newman LE, Shadel GS (2018). Mitohormesis in mice via sustained basal activation of mitochondrial and antioxidant signaling. Cell Metab.

[75] Kung-Chun Chiu D, Pui-Wah Tse A, Law CT, Ming-Jing Xu I, Lee D, Chen M, Kit-Ho Lai R, Wai-Hin Yuen V, Wing-Sum Cheu J, Wai-Hung Ho D, Wong CM, Zhang H, Oi-Lin Ng I, Chak-Lui Wong C (2019). Hypoxia regulates the mitochondrial activity of hepatocellular carcinoma cells through HIF/HEY1/PINK1 pathway. Cell Death Dis.

[76] Biala AK, Dhingra R, Kirshenbaum LA (2015). Mitochondrial dynamics: orchestrating the journey to advanced age. J Mol Cell Cardiol.

[77] Walters JW, Amos D, Ray K, Santanam N (2016). Mitochondrial redox status as a target for cardiovascular disease. Curr Opin Pharmacol.

[78] Bleier L, Wittig I, Heide H, Steger M, Brandt U, Drose S (2015). Generator-specific targets of mitochondrial reactive oxygen species. Free Radic Biol Med.

[79] Brand MD (2010). The sites and topology of mitochondrial superoxide production. Exp Gerontol.

[80] Lenaz G (2001). The mitochondrial production of reactive oxygen species: mechanisms and implications in human pathology. IUBMB Life.

[81] Wong HS, Dighe PA, Mezera V, Monternier PA, Brand MD (2017). Production of superoxide and hydrogen peroxide from specific mitochondrial sites under different bioenergetic conditions. J Biol Chem.

[82] Zhao RZ, Jiang S, Zhang L, Yu ZB (2019). Mitochondrial electron transport chain, ROS generation and uncoupling (review). Int J Mol Med.

[83] Badolia R, Ramadurai DKA, Abel ED, et al. The Role of Nonglycolytic Glucose Metabolism in Myocardial Recovery Upon Mechanical Unloading and Circulatory Support in Chronic Heart Failure. Circulation. 2020;142(3):259-74.10.1161/CIRCULATIONAHA.119.044452PMC738095632351122

[84] Zenkov NK, Kozhin PM, Chechushkov AV, Kandalintseva NV, Martinovich GG, Menshchikova EV (2020). Oxidative stress in aging. Adv Gerontol.

[85] Zhao J, Piao X, Wu Y, Liang S, Han F, Liang Q, Shao S, Zhao D (2020). Cepharanthine attenuates cerebral ischemia/reperfusion injury by reducing NLRP3 inflammasome-induced inflammation and oxidative stress via inhibiting 12/15-LOX signaling. Biomed Pharmacother.

[86] Bell EL, Chandel NS (2007). Mitochondrial oxygen sensing: regulation of hypoxia-inducible factor by mitochondrial generated reactive oxygen species. Essays Biochem.

[87] Grasso D, Zampieri LX, Capeloa T, Van de Velde JA, Sonveaux P (2020). Mitochondria in cancer. Cell Stress.

[88] Zhou J, Geng S, Ye W, Wang Q, Lou R, Yin Q, Du B, Yao H (2020). ROS-boosted photodynamic therapy against metastatic melanoma by inhibiting the activity of antioxidase and oxygen-producing nano-dopants. Pharmacol Res.

[89] Lai RK, Xu IM, Chiu DK, Tse AP, Wei LL, Law CT, Lee D, Wong CM, Wong MP, Ng IO, Wong CC (2016). NDUFA4L2 fine-tunes oxidative stress in hepatocellular carcinoma. Clin Cancer Res.

[90] Lucarelli G, Rutigliano M, Sallustio F, Ribatti D, Giglio A, Lepore Signorile M, Grossi V, Sanese P, Napoli A, Maiorano E, Bianchi C, Perego RA, Ferro M, Ranieri E, Serino G, Bell LN, Ditonno P, Simone C, Battaglia M (2018). Integrated multi-omics characterization reveals a distinctive metabolic signature and the role of NDUFA4L2 in promoting angiogenesis, chemoresistance, and mitochondrial dysfunction in clear cell renal cell carcinoma. Aging (Albany NY).

[91] Meng L, Yang X, Xie X, Wang M (2019). Mitochondrial NDUFA4L2 protein promotes the vitality of lung cancer cells by repressing oxidative stress. Thorac Cancer.

[92] Hinchliffe P, Sazanov LA (2005). Organization of iron-sulfur clusters in respiratory complex I. Science.

[93] Rouault TA, Tong WH. Iron-sulfur cluster biogenesis and human disease. Trends Genet. 2008;24:398–407.10.1016/j.tig.2008.05.008PMC257467218606475

[94] Neal CS, Michael MZ, Rawlings LH, Van der Hoek MB, Gleadle JM (2010). The VHL-dependent regulation of microRNAs in renal cancer. BMC Med.

[95] Chan SY, Zhang YY, Hemann C, Mahoney CE, Zweier JL, Loscalzo J (2009). MicroRNA-210 controls mitochondrial metabolism during hypoxia by repressing the iron-sulfur cluster assembly proteins ISCU1/2. Cell Metab.

[96] Fukuda R, Zhang H, Kim JW, Shimoda L, Dang CV, Semenza GL (2007). HIF-1 regulates cytochrome oxidase subunits to optimize efficiency of respiration in hypoxic cells. Cell.

[97] Sommer N, Hüttemann M, Pak O, Scheibe S, Knoepp F, Sinkler C, Malczyk M, Gierhardt M, Esfandiary A, Kraut S, Jonas F, Veith C, Aras S, Sydykov A, Alebrahimdehkordi N, Giehl K, Hecker M, Brandes RP, Seeger W, Grimminger F, Ghofrani HA, Schermuly RT, Grossman LI, Weissmann N (2017). Mitochondrial complex IV subunit 4 isoform 2 is essential for acute pulmonary oxygen sensing. Circ Res.

[98] Yoshida GJ, Azuma A, Miura Y, Orimo A. Activated Fibroblast Program Orchestrates Tumor Initiation and Progression; Molecular Mechanisms and the Associated Therapeutic Strategies. Int J Mol Sci. 2019;20(9):2256.10.3390/ijms20092256PMC653941431067787

[99] Yoshida GJ (2020). Regulation of heterogeneous cancer-associated fibroblasts: the molecular pathology of activated signaling pathways. J Exp Clin Cancer Res.

[100] Shida M, Kitajima Y, Nakamura J, Yanagihara K, Baba K, Wakiyama K, Noshiro H (2016). Impaired mitophagy activates mtROS/HIF-1alpha interplay and increases cancer aggressiveness in gastric cancer cells under hypoxia. Int J Oncol.

[101] Yoshida GJ (2017). Therapeutic strategies of drug repositioning targeting autophagy to induce cancer cell death: from pathophysiology to treatment. J Hematol Oncol.

[102] Chourasia AH, Macleod KF (2015). Tumor suppressor functions of BNIP3 and mitophagy. Autophagy.

[103] Zhang H, Bosch-Marce M, Shimoda LA, Tan YS, Baek JH, Wesley JB, Gonzalez FJ, Semenza GL (2008). Mitochondrial autophagy is an HIF-1-dependent adaptive metabolic response to hypoxia. J Biol Chem.

[104] Esteban-Martinez L, Boya P (2018). BNIP3L/NIX-dependent mitophagy regulates cell differentiation via metabolic reprogramming. Autophagy.

[105] Semenza GL (2003). Targeting HIF-1 for cancer therapy. Nat Rev Cancer.

[106] Akanji MA, Rotimi D, Adeyemi OS (2019). Hypoxia-inducible factors as an alternative source of treatment strategy for Cancer. Oxidative Med Cell Longev.

[107] Lang J, Zhao X, Wang X, Zhao Y, Li Y, Zhao R, Cheng K, Li Y, Han X, Zheng X, Qin H, Geranpayehvaghei M, Shi J, Anderson GJ, Hao J, Ren H, Nie G (2019). Targeted co-delivery of the Iron Chelator Deferoxamine and a HIF1alpha inhibitor impairs pancreatic tumor growth. ACS Nano.

[108] Liu YX, Feng JY, Sun MM, Liu BW, Yang G, Bu YN, Zhao M, Wang TJ, Zhang WY, Yuan HF, Zhang XD (2019). Aspirin inhibits the proliferation of hepatoma cells through controlling GLUT1-mediated glucose metabolism. Acta Pharmacol Sin.

[109] Cortes E, Lachowski D, Robinson B, et al. Tamoxifen mechanically reprograms the tumor microenvironment via HIF-1A and reduces cancer cell survival. EMBO Rep. 2019;20(1):e46557.10.15252/embr.201846557PMC632238830538116

[110] Guimaraes TA, Farias LC, Santos ES, de Carvalho Fraga CA, Orsini LA, de Freitas Teles L, Feltenberger JD, de Jesus SF, de Souza MG, Santos SH, de Paula AM, Gomez RS, Guimaraes AL (2016). Metformin increases PDH and suppresses HIF-1alpha under hypoxic conditions and induces cell death in oral squamous cell carcinoma. Oncotarget.

[111] Lu H, Li X, Luo Z, Liu J, Fan Z (2013). Cetuximab reverses the Warburg effect by inhibiting HIF-1-regulated LDH-A. Mol Cancer Ther.

[112] Fumarola C, Cretella D, La Monica S, Bonelli MA, Alfieri R, Caffarra C, Quaini F, Madeddu D, Falco A, Cavazzoni A, Digiacomo G, Mazzaschi G, Vivo V, Barocelli E, Tiseo M, Petronini PG, Ardizzoni A (2017). Enhancement of the anti-tumor activity of FGFR1 inhibition in squamous cell lung cancer by targeting downstream signaling involved in glucose metabolism. Oncotarget.

[113] Ashburn TT, Thor KB (2004). Drug repositioning: identifying and developing new uses for existing drugs. Nat Rev Drug Discov.

[114] Shukla SK, Purohit V, Mehla K, Gunda V, Chaika NV, Vernucci E, King RJ, Abrego J, Goode GD, Dasgupta A, Illies AL, Gebregiworgis T, Dai B, Augustine JJ, Murthy D, Attri KS, Mashadova O, Grandgenett PM, Powers R, Ly QP, Lazenby AJ, Grem JL, Yu F, Mates JM, Asara JM, Kim JW, Hankins JH, Weekes C, Hollingsworth MA, Serkova NJ, Sasson AR, Fleming JB, Oliveto JM, Lyssiotis CA, Cantley LC, Berim L, Singh PK (2017). MUC1 and HIF-1alpha Signaling Crosstalk Induces Anabolic Glucose Metabolism to Impart Gemcitabine Resistance to Pancreatic Cancer. Cancer Cell.

[115] Kim EH, Ko HY, Yu AR, et al. Inhibition of HIF-1α by Atorvastatin During 131I-RTX Therapy in Burkitt's Lymphoma Model. Cancers (Basel). 2020;12(5):1203.10.3390/cancers12051203PMC728165532403237

[116] Wei TT, Lin YT, Tang SP, Luo CK, Tsai CT, Shun CT, Chen CC (2020). Metabolic targeting of HIF-1alpha potentiates the therapeutic efficacy of oxaliplatin in colorectal cancer. Oncogene.

[117] Lee JW, Yang DH, Park S, Han HK, Park JW, Kim BY, Um SH, Moon EY (2018). Trichostatin a resistance is facilitated by HIF-1alpha acetylation in HeLa human cervical cancer cells under normoxic conditions. Oncotarget.

[118] Choi YJ, Shin HW, Chun YS, Leutou AS, Son BW, Park JW (2016). Diacetoxyscirpenol as a new anticancer agent to target hypoxia-inducible factor 1. Oncotarget.

[119] Wang J, Li G, Wang Y, Tang S, Sun X, Feng X, Li Y, Bao G, Li P, Mao X, Wang M, Liu P (2015). Suppression of tumor angiogenesis by metformin treatment via a mechanism linked to targeting of HER2/HIF-1alpha/VEGF secretion axis. Oncotarget.

[120] Tyszka-Czochara M, Bukowska-Strakova K, Kocemba-Pilarczyk KA, Majka M. Caffeic Acid Targets AMPK Signaling and Regulates Tricarboxylic Acid Cycle Anaplerosis while Metformin Downregulates HIF-1α-Induced Glycolytic Enzymes in Human Cervical Squamous Cell Carcinoma Lines. Nutrients. 2018;10(7):841.10.3390/nu10070841PMC607380529958416

[121] Chen HF, Wu LX, Li XF, Zhu YC, Wang WX, Xu CW, Huang ZZ, Du KQ (2019). Ginsenoside compound K inhibits growth of lung cancer cells via HIF-1alpha-mediated glucose metabolism. Cell Mol Biol (Noisy-le-grand).

[122] Lam W, Bussom S, Cheng YC (2009). Effect of hypoxia on the expression of phosphoglycerate kinase and antitumor activity of troxacitabine and gemcitabine in non-small cell lung carcinoma. Mol Cancer Ther.

